# Identification of novel candidate indicators for assessing zinc status during pregnancy in mice from microarray data

**DOI:** 10.1186/s40360-019-0288-8

**Published:** 2019-02-15

**Authors:** Wan Xu, Hongyan Wu, Lixin Shang

**Affiliations:** 1 The Fourth Military Medical University, Xi’an, Shaanxi Province, 710032 China; 2 Department of Obstetrics and Gynecology, PLA Army General Hospital, No.5 Nanmencang, Dongcheng District, Beijing, 100700 China

**Keywords:** Zinc deficiency, Differentially expressed genes, Protein-protein interaction, Module

## Abstract

**Background:**

This study aimed to identify potential zinc status indicators and to clarify the mechanisms underlying zinc deficiency-induced organ damage and mortality in mice.

**Methods:**

The dataset GSE97112, including placental tissues of mice fed diets containing normal and low concentrations of zinc, was downloaded and preprocessed. Differentially expressed genes (DEGs) were calculated and identified for zinc deficiency-related gene clusters by using the weighed gene co-expression network analysis (WGCNA) algorithm. The Gene Ontology (GO)-Biological Process (BP) and KEGG pathway of genes in the zinc deficiency-related WGCNA modules were analyzed, and the protein-protein interaction (PPI) network was constructed. In addition, modules of the PPI network were identified, and transcription factors (TFs) and miRNAs regulating DEGs were predicted. Finally, drug-gene interactions were selected.

**Results:**

A total of 1055 DEGs containing 586 up- and 469 down-regulated genes were obtained. Three modules based on WGCNA had high correlation with degree of zinc deficiency. Annexin A1 (*ANXA1*), C-C motif chemokine receptor 3 (*CCR3*), C-X-C motif chemokine receptor 2 (*CXCR2*), and interleukin 2 (*IL-2*) were hub nodes in the PPI network. Three modules in the PPI network were identified, including module 1 associated with olfactory conduction and module 2 associated with inflammatory response. *ANXA1*, *CCR3,* and *IL*-2 were regulated by TFs. In addition, *CXCR2*, *ANXA*, and *IL*-2 were drug targets.

**Conclusion:**

*CXCR2*, *ANXA1,* and *CCR3* as well as olfactory receptor-related genes (proteins) may be used as biomarkers to assess zinc status in mice.

## Background

Zinc as an important metal is involved in numerous metabolic processes. Inadequate zinc intake is highly prevalent worldwide. Wessells and Brown have estimated that at least 17% of the world’s population suffers from inadequate zinc intake [1]. Zinc is also an indispensable trace element during pregnancy, and zinc deficiency because of maternal nutritional deficiency can result in severe fetal growth restriction [2]. Severe zinc deficiency in pregnancy can result in increased fetal loss and high rates of congenital malformations in several organs of surviving fetuses [3, 4]. Furthermore, inadequate zinc intake is thought to be a leading cause of infant mortality [5].

Plasma zinc is widely used as a biomarker of zinc status [6, 7]. However, decrease of serum zinc concentration is only detectable after long-term or severe depletion, making serum zinc an unreliable biomarker of zinc status [6]. Novel zinc biomarkers, such as the erythrocyte linoleic acid:dihomo-γ-linolenic acid ratio, negatively correlate with plasma Zn status [8–10]. However, there is no valid, sensitive, and reliable biomarker for zinc deficiency, particularly for marginal zinc deficiency. Previous studies have shown that changes in expression of several zinc transporters (ZnTs) influence zinc homeostasis and metabolism and subsequently change zinc status [11–14]. Moreover, dysregulation of other molecules, such as cytokines [15], ProSAP/Shank family members [16], antioxidant enzymes, and heat shock proteins [17] are associated with zinc status. Therefore, abnormal expression of genes could be a potential biomarker for zinc deficiency during pregnancy in the placenta.

In this study, microarray technology and bioinformatics methods were used to identify genes whose expression was influenced by zinc deficiency using the microarray data GSE97112 [18], which has been used to illustrate the relationship between abnormal gene expression and mean arterial pressure changes during gestation in mice. A systematic bioinformatics analysis of GSE97112 was conducted in the study. The results may help to identify potential zinc status indicators and to clarify the mechanisms underlying zinc deficiency-induced organ damage and mortality.

## Materials and methods

### Data downloading and pre-processing

The original CEL file of the dataset GSE97112 [18] was downloaded from Gene Expression Omnibus (GEO, http://www.ncbi.nlm.nih.gov/geo/). The samples were placental tissues of seven-week-old C57Bl/6J female mice fed a diet containing different concentrations of zinc from 6 weeks prior to gestation to the conclusion of experiments. The animals were divided into the following groups: control (40 mg/kg zinc, 20 cases) and zinc deficient (10 mg/kg zinc, 12 cases). The chip platform was Affymetrix Mouse Gene 2.1 ST Array, and the data were downloaded in June 2018.

The raw data were read using the R 3.4.0 extension package oligo [19] (Version 1.44.0, http://www.bioconductor.org/packages/release/bioc/html/oligo.html), preprocessed using the robust multi-array average (RMA) method [20, 21] for data normalization, and were annotated using R package mogene21sttranscriptcluster.db (version 8.7.0, http://bioconductor.org/packages/release/data/annotation/html/mogene21sttranscriptcluster.db.html) to remove probes that did not match the transcript (Gene symbol). For different probes mapped to the same gene, the mean value of the different probes was taken as the final expression value of the gene.

### Differential expression analysis of genes

Differentially expressed genes (DEGs) were calculated using the empirical Bayes linear model in the R package limma [22] (Version 3.32.5, http://bioconductor.org/packages/release/bioc/html/limma.html) for the *P* value of all genes. The significance threshold for DEGs was a *P* value < 0.05.

### Disease related modules and genes by weighed gene co-expression network analysis (WGCNA)

The WGCNA algorithm was used to discover gene clusters (or modules) in high-throughput data that were highly correlated with the sample phenotype. Modular characteristic genes in these modules were summarized, and the modules that were significantly associated with the phenotype were further evaluated.

The R package WGCNA [23] (Version 1.61, https://cran.r-project.org/web/packages/WGCNA/) was used to identify gene sets that were significantly associated with zinc deficiency from DEGs. By setting a series of soft-thresholding power values, the correlation coefficient and the average connection degree of the connection degrees k and p(k) under each power value were calculated. The threshold was a correlation coefficient > 0.85. Based on clustering and dynamic pruning, the highly correlated genes were aggregated into modules. Finally, the WGCNA modules associated with the disease (zinc deficiency) were identified.

### Functional enrichment analysis

The commonly used enrichment analysis tool Database for Annotation Visualization and Integrated Discovery (DAVID) [24] (version 6.8, https://david-d.ncifcrf.gov/) that was based on hypergeometric distribution was used to analyze the Gene Ontology (GO)-Biological Process (BP) [25] and KEGG pathway [26] of genes in the zinc deficiency-related WGCNA modules. Results with a *P* value < 0.05 were considered to be significantly enriched.

### Protein-protein interaction (PPI) network construction

PPI network is available for identification of cellular functions of proteins in various organisms [27], facilitating to identification of key proteins associated with zinc deficiency. The interactions between gene-encoded proteins in the disease-related WGCNA modules were predicted based on the STRING [28] (version: 10.0, http://www.string-db.org/) database. The input gene set was the genes in WGCNA modules which were significantly associated with zinc deficiency. The species was *Mus musculus*, and the parameter of PPI score was set to 0.7 (high confidence). Protein nodes were all included in the disease-related WGCNA modules.

After obtaining the PPI relationship, a network diagram was constructed using Cytoscape software [29]. Then the CytoNCA [30] plugin (version 2.1.6, http://apps.cytoscape.org/apps/cytonca) was used to analyze the topological properties of the network without weighting. The Degree Centrality (DC), Betweenness Centrality (BC), and Closeness Centrality (CC) were obtained and nodes were ranked based on topological properties of the network. The most important node of the PPI network involved in protein interaction was identified and designated as the hub protein.

### Modules of the PPI network

Using the MCODE plugin [31] of Cytoscape software, the function module was identified, and the relationship between network topology and network components was obtained using default parameters (Degree Cutoff = 2, Node Score Cutoff = 0.2, K-core = 2, Max.Depth = 100). DAVID was also used to perform GO-BP and KEGG pathway enrichment analysis for genes in modules with threshold scores > 4.

### Predicting transcription factors (TFs) and miRNAs regulating DEGs

TFs and miRNAs can play important regulatory roles in gene expression. To better understand the regulatory mechanism affected by zinc deficiency, TFs and miRNAs that could regulate key genes/proteins associated with zinc deficiency were predicted. In this study, the WebGestalt GAST [32] (http://www.webgestalt.org/option.php) tool was used for prediction of miRNA and TFs in the PPI network. The Overrepresentation Enrichment Analysis (ORA) enrichment method was used to predict miRNA-target and TF-target with the minimum enriched gene number of 5.

### Therapeutic drug prediction

The Drug-Gene Interaction database (DGIdb) database [33] (http://www.dgidb.org/) was used to predict genes targeted by the therapeutic drug, which will provide a new perspective for designing effective targeted drugs for prevention of zinc deficiency. Literature-supported drug-gene interactions were selected to construct network maps.

## Results

### Differential expression analysis

After data preprocessing, a gene expression matrix containing 32 samples and 23,992 genes was obtained. The distribution of gene expression levels before and after standardization showed that the gene expression levels between samples were nearly a straight line after normalization, which was suitable for further analysis.

Based on the determined thresholds, 1055 DEGs containing 586 up- and 469 down-regulated genes were obtained. The bidirectional clustering heat map of DEGs was shown in Fig. 1. The results showed that DEGs could clearly distinguish the samples according to the zinc concentration, indicating that these genes showed significant changes following treatment with different concentrations of zinc, which suggested that these were genes potentially associated with degree of zinc deficiency.

**Fig. 1:** Heatmap of differentially expressed genes (DEGs) in 12 zinc deficient samples and 20 control samples from placenta tissues of mice. Red and green represent high and low expression, respectively, and white refers to missing expression values

### Modules and genes screened by WGCNA

To further screen genes associated with zinc deficiency, we performed a WGCNA analysis of the differential gene expression matrices obtained in the previous step. According to the method, the power value when the correlation coefficient squared value of connection degree k and p(k) for the first time to reach 0.85 (green line) were selected, that was, power = 7; under this power parameter, the average connectivity of the constructed co-expressing network nodes was 0.875, as shown in Fig. 2 (right). In addition, k was negatively correlated with p(k), indicating that the selected power value could be used for establishing a gene-scale network.

**Fig. 2:** Results of the weighed gene co-expression network analysis (WGCNA) module and trait correlation analysis. Left panel: Trait-related modules were mined based on the correlation between traits and module eigenvector genes and *p* values. Right panel: the mean of correlation coefficients between traits and gene expression levels in each module as the significant of the trait in the module

Based on clustering and dynamic pruning, 1055 highly correlated genes were clustered into 5 modules, where the grey module was a collection of genes that could not be aggregated to other modules. The 5 modules were clustered when the correlation coefficient was greater than 0.8, that was, the module with the dissimilarity coefficient less than 0.2 was merged. As a result, 4 WGCNA modules were constructed.

Two methods were used to mine modules related to degree of zinc deficiency: the correlation between each module’s feature vector gene and the degree of zinc deficiency was calculated; the correlation between the traits and the expression of each gene in each module as the significance of the trait in the module, with greater significance signifying greater relevance between the module and the trait (Fig. 2, left). As a result, three modules (except for the gray) had high correlation with degree of zinc deficiency (Fig. 2, right). The yellow module contained 160 genes including 81 up-regulated and 79 down-regulated genes. The blue module contained 469 differential genes, of which 292 were up-regulated and 177 were down-regulated. The brown module contained 185 genes, of which 104 were up-regulated and 81 were down-regulated.

### Functional terms and pathways enriched by DEGs in WGCNA modules

GO-BP enrichment analysis and KEGG pathway enrichment analysis results showed that the genes in the blue module were mainly associated with chloroplast transmembrane transport and cell meiosis. The genes in the brown module were mainly enriched in GO-BP terms of transcriptional regulation, and multicellular organism development, as well as pathways related to glycerophospholipid metabolism, and the transcription factor regulatory of the FOXO family. The yellow module gene in GO-BP terms was related to negative regulation of myoblast differentiation, multicellular organism development, and cell differentiation, as well as pathways of cytokines, and transport and catabolic of peroxidases.

### PPI network constructed by DEGs in WGCNA modules

PPI analysis of DEGs in three WGCNA modules was performed. Two hundred forty-six PPI relationship pairs for 150 DEGs were obtained. Among these, 75 genes were up-regulated and 75 genes were down-regulated. The topological properties of the PPI network were analyzed, and the DC, BC, and CC scores of the top 30 nodes were shown in Table 1. DEGs of Annexin A1 (*ANXA1*), C-C motif chemokine receptor 3 (*CCR3*), C-X-C motif chemokine receptor 2 (*CXCR2*), dynein light chain, LC8-type 2 (*DYNLL2*), interleukin 2 (*IL*-2), SEC13 homolog, nuclear pore and COPII coat complex component (*SEC13*), and transforming growth factor beta 1 (*TGFB1*) were in three ranks, which might represent hub nodes in the network.

**Table 1:** Top 30 nodes ranked by Degree Centrality (DC), Betweenness Centrality (BC), and Closeness Centrality (CC) in the protein-protein interaction network

Genes	Degree	Genes	Betweenness	Genes	Closeness
Olfr316	13	IL-2	1952.8	Cd247	1.11E-02
Olfr1392	13	Sec13	1905.2	H2-M10.1	1.11E-02
Olfr555	13	H2-M10.1	1491.2	Sec13	1.11E-02
Olfr308	13	Tmed2	1216.2	Cd8b1	1.11E-02
Olfr384	13	Cd247	1116.2	IL-2	1.11E-02
Olfr323	13	Ccr3	1109	Tmed2	1.11E-02
Olfr790	13	Seh1l	1020	Shc3	1.11E-02
Olfr1090	13	Casc3	936	Seh1l	1.11E-02
Olfr804	13	Dynll2	888	Ccr3	1.11E-02
Olfr365	13	Cd8b1	624.6	Sec22b	1.11E-02
Olfr646	13	Shc3	591.8	Mios	1.10E-02
Olfr872	13	Tgfb1	538	Tgfb1	1.10E-02
Olfr734	13	Notch1	470	Ntrk2	1.10E-02
Olfr171	13	Exosc3	462	Dvl3	1.10E-02
Anxa1	10	Dvl3	418.8	Notch1	1.10E-02
IL-2	9	Prkag2	354	Serpinb6b	1.10E-02
Ccr3	9	Anxa1	348	Serpinb5	1.10E-02
Cxcr2	8	Ntrk2	324.8	Serpinb9c	1.10E-02
Insl5	7	Egf	266.6	Hand2	1.10E-02
Npw	7	Utp18	236	Il18	1.10E-02
Gal	7	Rpl28	215.3	Dynll2	1.10E-02
S1pr4	7	Rpl18a	215.3	Pdgfra	1.10E-02
P2ry13	7	Rpl35a	215.3	Casc3	1.10E-02
Dynll2	6	Pdgfra	187.2	Egf	1.10E-02
Abcg3	5	Tfrc	120	Hgf	1.10E-02
Exosc3	5	Wnt3a	120	Gfra1	1.10E-02
Tgfb1	5	Hgf	30.6	Anxa1	1.10E-02
Sec13	5	Abcg3	20	Cxcr2	1.10E-02
Rpl28	5	Atm	12	Insl5	1.10E-02
Rpl18a	5	Cxcr2	9	Npw	1.10E-02

In addition, 7 modules were identified from the PPI network. As shown in Fig. 3, there were 3 modules with score > 4, where module 1 contained 8 up-regulated genes and 6 down-regulated genes, all of which were olfactory receptor-related genes. Module 2 included 4 up-regulated genes and 4 down-regulated genes, including *ANXA1*, *CCR3* and *CXCR2*. Module 3 contained 4 up-regulated genes and 2 down-regulated genes.

**Fig. 3:** Three modules with score > 4 identified from the protein-protein interaction (PPI) network. Red circles indicate up-regulated genes, and green circles represent down-regulated genes. The edges refer to the interactions between two nodes

The GO-BP and KEGG pathway analyses were performed on the genes grouped in the three modules. The results in Table 2 showed that module 1 was mainly involved in olfactory conduction and protein-coupled receptor signaling pathways. Module 2 was mainly enriched in BP terms related to signal transduction, inflammatory response, and angiogenesis. Module 3 was mainly involved in translation, rRNA, and ribosome related pathways.

**Table 2:** The Gene Ontology (GO)-Biological Process (BP) and KEGG pathway analyses of genes of the three modules from the protein-protein interaction network

Module	Category	Term	Count	P Value	Genes
Module 1	GO_BP	GO:0007608~sensory perception of smell	14	2.41E-16	OLFR872/OLFR323/OLFR734/OLFR308/OLFR646/OLFR555/OLFR316/OLFR384/OLFR804/OLFR171/OLFR365/OLFR1392/OLFR790/OLFR1090
	GO_BP	GO:0007186~G-protein coupled receptor signaling pathway	14	4.50E-14	OLFR872/OLFR323/OLFR734/OLFR308/OLFR646/OLFR555/OLFR316/OLFR384/OLFR804/OLFR171/OLFR365/OLFR1392/OLFR790/OLFR1090
	GO_BP	GO:0050907~detection of chemical stimulus involved in sensory perception	3	9.28E-03	OLFR734/OLFR384/OLFR365
	KEGG_PATHWAY	mmu04740:Olfactory transduction	12	3.84E-10	OLFR872/OLFR323/OLFR734/OLFR308/OLFR646/OLFR555/OLFR384/OLFR171/OLFR365/OLFR1392/OLFR790/OLFR1090
Module 2	GO_BP	GO:0007165~signal transduction	5	6.82E-04	P2RY13/CCR3/S1PR4/ANXA1/CXCR2
	GO_BP	GO:0007186~G-protein coupled receptor signaling pathway	5	2.19E-03	P2RY13/CCR3/NPW/S1PR4/CXCR2
	GO_BP	GO:0006954~inflammatory response	3	7.11E-03	CCR3/ANXA1/GAL
	GO_BP	GO:0007631~feeding behavior	2	1.31E-02	NPW/GAL
	GO_BP	GO:0006935~chemotaxis	2	4.48E-02	CCR3/CXCR2
	GO_BP	GO:0045766~positive regulation of angiogenesis	2	4.59E-02	CCR3/CXCR2
Module 3	GO_BP	GO:0006412~translation	3	2.86E-03	RPL35A/RPL18A/RPL28
	GO_BP	GO:0006364~rRNA processing	2	2.76E-02	RPL35A/EXOSC3
	KEGG_PATHWAY	mmu03010:Ribosome	3	2.05E-03	RPL35A/RPL18A/RPL28

### DEGs were regulated by miRNAs and TFs

Based on Webgestalt prediction, 303 TF-Target relationship pairs were obtained, including 35 TFs and 85 target genes. Forty-one miRNA-target relationship pairs were obtained, including 5 miRNAs and 23 target genes. As shown in Fig. 4, The TFs with the highest number of target genes were summarized. Calcium voltage-gated channel subunit alpha1 a (*CACNA1a*), *CACNA1d*, and mitogen-activated protein kinase kinase 6 (*MAP2K6*) were simultaneously regulated by multiple TFs and miRNAs. According to the results of functional and pathway analysis, these genes were involved in solute transmembrane transport, positive regulation of apoptosis, multicellular organism development, and biological process of MAPK activity activation. The hub proteins *ANXA1*, *CCR3*, *DYNLL2*, *IL*-2, *SEC13*, and *TGFB1* in the above PPI network were regulated by the TFs of P53/TATA, CCAAT/enhancer binding protein (CEBP), Paired Box 3 (PAX3), Nuclear Factor Kappa B (NFKB)/E74 like ETS transcription factor 2 (ELF2)/heat-shock transcription factor 2 (HSF2), GA-binding protein (GABP), and ELF1/myeloid zinc finger gene 1 (MZF1), respectively.

**Fig. 4:** The transcription factor (TF)-miRNA-target regulatory network. Red circles indicate up-regulated genes, green circles indicate down-regulated genes, yellow triangles represent predicted miRNAs, purple diamonds indicate predicted TFs (only TOP5 with higher number of target genes than others), red arrows indicate miRNA-regulated target genes, and gray arrows indicate target genes regulated by TFs

### Therapeutic drug prediction

Based on the DGIdb database, the interaction network diagram of drug-gene interactions was constructed (Fig. 5). Eighty-three drug-target relationship pairs, including 4 DEGs and 80 interaction drugs were identified. The 4 DEGs were *CXCR2*, *ANXA*, *TGFB1,* and *IL*-2.

**Fig. 5:** The drug-target gene interaction network. Blue circles represent the key genes, and the white hexagon represents the predicted drug interactions

## Discussion

Zinc is reported to exert antioxidant activity through guarding sulfhydryl groups and stabilization of cell membranes, and it may play a key role in modulating cell cycle and apoptosis [34, 35]. Two zinc transporter families, ZnTs and Zrt-, Irt-related proteins (ZIPs) are shown to function in zinc mobilization across biological membranes [14]. For instance, ZnT 1 is shown to play a key role in zinc homeostasis in adult mice via modulating the transport of maternal zinc into the embryonic environment, and deletion of the Zinc Transporter 1 gene in mice may result in embryonic lethal [36]. ZIP8 can function indispensable effects on both multiple-organ organogenesis and hematopoiesis during early embryogenesis in mice [37]. Moreover, Zinc deficiency during pregnancy is harmful for both the mother and the fetus [38], which is considered as a risk factor for adverse pregnancy outcomes and preterm delivery [39]. As such, effective monitoring for zinc deficiency is very important. In this study, some potential biomarkers for zinc deficiency during pregnancy in the placentas of mice were identified.

Zinc is essential for immunity, oxidative stress, and chronic inflammatory response [40]. Zinc deficiency is involved in immune dysfunction and systemic inflammation [41] and was found to exert a significant influence on the outcome of inflammatory diseases, such as inflammatory bowel disease [42]. Moreover, maternal zinc supplementation is found to impact beneficial effects on neonatal immune status and infant morbidity from infectious diseases [43]. This study revealed that *CXCR2*, *CCR3*, *ANXA1*, and *IL*-2 were hub nodes in the PPI network and were regulated by TFs. The chemokine receptor *CXCR2,* involving in the innate immune system, is a receptor for interleukin 8 (IL-8). It mediates neutrophil migration to sites of inflammation and angiogenic effects [44]. *CCR3* encodes a receptor for C-C type chemokines which contributes to accumulation and activation of eosinophils and inflammatory cells [45]. *IL*-2 regulates proliferation of T and B lymphocytes and plays an essential role in the immune response [46]. *ANXA1* has anti-inflammatory activity and is important for innate immune response [47]. The functional enrichment results confirmed the relationship between three genes and immune response. Prasad et al. suggested that *IL*-2 and *IL*-2 receptors were down-regulated during zinc deficiency [48]. However, there is no evidence of relationship of abnormal expression of the three genes (*CXCR2*, *CCR3* and *ANXA1*) and zinc deficiency. Therefore, *CXCR2*, *ANXA1,* and *CCR3* would be potential biomarkers for zinc deficiency in mice. In addition, therapeutic drug prediction indicated that *CXCR2* and *ANXA1* may be targets of drugs, suggesting these two genes may be implicated as therapeutic targets to reduce risk of zinc deficiency. Notably, there is no currently available information that supports the routine use of zinc supplementation on improving pregnancy outcome [43]. Moreover, it is challenging to the implementation of targeted interventions for reducing the adverse effects of zinc deficiency through therapeutic and preventive supplementation, fortification, and biofortification [39]. Given the side effects of many drugs, especially to the fetus, the best option is to consume dietary zinc (abundant in meat and beans) for improving mild zinc deficiency, rather than using medicines.

In addition, it is noted that the PPI network module 1 was composed entirely olfactory receptor-related genes. Zinc is highly concentrated in the olfactory bulb of the brain and is important for embryonic neural development of the olfactory system [49, 50]. In recent years, zinc research has mainly focused on zinc metal nanoparticles, which could enhance odorant responses of olfactory receptor neurons [51]. These results suggested that zinc deficiency may affect development of the central olfactory system. Therefore, these genes may be used as gene biomarkers for zinc deficiency in pregnant mice.

However, the nutrients in mouse diet were largely unknown because the microarray data were downloaded from a public database, and the presence of other metals such as cadmium in the diet that could compete with Zn absorption was unknown. Moreover, we did not perform experiments or analyze another appropriate dataset to validate the differential expression of key genes associated with zinc deficiency. Furthermore, it is hard to extrapolate mouse data to human biochemistry, as the genetic origin of the placenta differs between mice and humans. Further experiments using human samples will provide stronger evidence for clinical guidance.

## Conclusion

Embryonic olfactory system development, immune dysfunction, and systemic inflammation may be disturbed by zinc deficiency. Expression levels of *CXCR2*, *ANXA1,* and *CCR3*, as well as olfactory receptor-related genes (proteins) may be used as biomarker to assess zinc status in mice.

## Abbreviations

*ANXA1*: Annexin A1
BC: Betweenness Centrality
BP: Biological Process
CC: Closeness Centrality
*CCR3*: C-C motif chemokine receptor 3
CEBP: CCAAT/enhancer binding protein
*CXCR2*: C-X-C motif chemokine receptor 2
DC: Degree Centrality
DEGs: Differentially expressed genes
*DYNLL2*: Dynein light chain, LC8-type 2
ELF2: ETS transcription factor 2
GABP: GA-binding protein
GO: Gene Ontology
HSF2: Heat-shock transcription factor 2
*IL-2*: Interleukin 2
IL-8: Interleukin 8
*MAP2K6*: Mitogen-activated protein kinase kinase 6
MZF1: Myeloid zinc finger gene 1
NFKB: Nuclear Factor Kappa B
ORA: Overrepresentation Enrichment Analysis
PAX3: Paired Box 3
PPI: Protein-protein interaction
TF: Transcription factor
*TGFB1*: Transforming growth factor beta 1
WGCNA: Weighted gene co-expression network analysis
ZIPs: Zrt-, Irt-related proteins
ZnTs: Zn transporters

## References

[1] Wessells KR, Brown KH (2012). Estimating the global prevalence of zinc deficiency: results based on zinc availability in national food supplies and the prevalence of stunting. PLoS One.

[2] Wang H, Hu YF, Hao JH, Chen YH, Su PY, Wang Y, Yu Z, Fu L, Xu YY, Zhang C (2015). Maternal zinc deficiency during pregnancy elevates the risks of fetal growth restriction: a population-based birth cohort study. Sci Rep.

[3] Hurley LS, Mutch PB (1973). Prenatal and postnatal development after transitory gestational zinc deficiency in rats. J Nutr.

[4] Uriu-Adams JY, Keen CL (2010). Zinc and reproduction: effects of zinc deficiency on prenatal and early postnatal development. Birth Defects Research Part B: Developmental and Reproductive Toxicology.

[5] Wadhwa N, Basnet S, Natchu UCM, Shrestha LP, Bhatnagar S, Sommerfelt H, Strand TA, Ramji S, Aggarwal KC, Chellani H (2017). Zinc as an adjunct treatment for reducing case fatality due to clinical severe infection in young infants: study protocol for a randomized controlled trial. Bmc Pharmacology & Toxicology.

[6] Lowe NM, Fekete K, Decsi T, Fairweathertait SJ, Harvey LJ, Casgrain A, Hooper L (2009). Methods of assessment of zinc status in humans: a systematic review. Am J Clin Nutr.

[7] Soltan MH, Jenkins DM (2010). Maternal and fetal plasma zinc concentration and fetal abnormality. British Journal of Obstetrics & Gynaecology.

[8] Reed S, Qin X, Ranressler R, Brenna JT, Glahn RP, Tako E (2014). Dietary zinc deficiency affects blood linoleic acid: Dihomo-γ-linolenic acid (LA:DGLA) ratio; a sensitive physiological marker of zinc status in vivo (Gallus gallus). Nutrients.

[9] Holen T, Norheim F, Gundersen TE, Mitry P, Linseisen J, Iversen PO, Drevon CA (2016). Biomarkers for nutrient intake with focus on alternative sampling techniques. Genes Nutr.

[10] Knez M, Stangoulis JCR, Zec M, Debeljak-Martacic J, Pavlovic Z, Gurinovic M, Glibetic M (2016). An initial evaluation of newly proposed biomarker of zinc status in humans - linoleic acid: dihomo-γ-linolenic acid (LA:DGLA) ratio. Clinical Nutrition Espen.

[11] Andree KB, Kim J, Kirschke CP, Gregg JP, Paik H, Joung H, Woodhouse L, King JC, Huang L (2004). Investigation of lymphocyte gene expression for use as biomarkers for zinc status in humans. J Nutr.

[12] Dufner-Beattie J, Huang ZL, Geiser J, Xu W, Andrews GK (2010). Mouse ZIP1 and ZIP3 genes together are essential for adaptation to dietary zinc deficiency during pregnancy. Genesis.

[13] Alsufiani HMA (2016). Zinc intake, zinc status and expression of zinc transporter genes in younger and older Saudi adults.

[14] Kambe T, Tsuji T, Hashimoto A, Itsumura N (2015). The physiological, biochemical, and molecular roles of zinc transporters in zinc homeostasis and metabolism. Physiol Rev.

[15] Aydemir TB, Blanchard RK, Cousins RJ (2006). Zinc supplementation of young men alters metallothionein, zinc transporter, and cytokine gene expression in leukocyte populations. Proc Natl Acad Sci U S A.

[16] Grabrucker S, Jannetti L, Eckert M, Gaub S, Chhabra R, Pfaender S, Mangus K, Reddy PP, Rankovic V, Schmeisser MJ (2014). Zinc deficiency dysregulates the synaptic ProSAP/shank scaffold and might contribute to autism spectrum disorders. Brain A Journal of Neurology.

[17] Wu C, Zhang W, Mai K, Xu W, Zhong X (2011). Effects of dietary zinc on gene expression of antioxidant enzymes and heat shock proteins in hepatopancreas of abalone Haliotis discus hannai. Comp Biochem Physiol C Toxicol Pharmacol.

[18] Wilson RL, Leemaqz SY, Goh Z, Mcaninch D, Jankovickarasoulos T, Leghi GE, Phillips JA, Colafella KM, Tran C, O’Leary S (2017). Zinc is a critical regulator of placental morphogenesis and maternal hemodynamics during pregnancy in mice. Sci Rep.

[19] Gautier L, Cope L, Bolstad BM, Irizarry RA (2004). Affy--analysis of Affymetrix GeneChip data at the probe level. Bioinformatics.

[20] Bolstad BM, Irizarry RA, Astrand M, Speed TP (2003). A comparison of normalization methods for high density oligonucleotide array data based on variance and bias. Bioinformatics.

[21] Irizarry RA, Hobbs B, Collin F, Beazer-Barclay YD, Antonellis KJ, Scherf U, Speed TP (2003). Exploration, normalization, and summaries of high density oligonucleotide array probe level data. Biostatistics.

[22] Smyth GK. Limma: linear models for microarray data, in bioinformatics and computational biology solutions using R and Bioconductor. Springer. 2005:397–420.

[23] Langfelder P, Horvath S (2008). WGCNA: an R package for weighted correlation network analysis. BMC bioinformatics.

[24] Huang DW, Sherman BT, Lempicki RA (2008). Systematic and integrative analysis of large gene lists using DAVID bioinformatics resources. Nat Protocols.

[25] Ashburner M, Ball CA, Blake JA, Botstein D, Butler H, Cherry JM, Davis AP, Dolinski K, Dwight SS, Eppig JT (2000). Gene ontology: tool for the unification of biology. Nat Genet.

[26] Kanehisa M, Goto S (2000). KEGG: Kyoto encyclopedia of genes and genomes. Nucleic Acids Res.

[27] Patil A, Nakamura H (2005). Filtering high-throughput protein-protein interaction data using a combination of genomic features. BMC bioinformatics.

[28] Szklarczyk D, Franceschini A, Wyder S, Forslund K, Heller D, Huerta-Cepas J, Simonovic M, Roth A, Santos A, Tsafou KP. STRING v10: protein–protein interaction networks, integrated over the tree of life. Nucleic acids research. 2014; gku1003.10.1093/nar/gku1003PMC438387425352553

[29] Shannon P, Markiel A, Ozier O, Baliga NS, Wang JT, Ramage D, Amin N, Schwikowski B, Ideker T (2003). Cytoscape: a software environment for integrated models of biomolecular interaction networks. Genome Res.

[30] Yu Tang ML, Wang J, Pan Y, Wu f-X (2014). CytoNCA: a cytoscape plugin for centrality analysis and evaluation of biological networks. BioSystems.

[31] Bader GDHC. An automated method for finding molecular complexes in large protein interaction networks. BMC Bioinformatics. 2003;13.10.1186/1471-2105-4-2PMC14934612525261

[32] Wang J, Duncan DT, Shi Z, Zhang B: WEB-based GEne SeT AnaLysis Toolkit (WebGestalt): update 2013. In Design, Automation & Test in Europe Conference & Exhibition 2013: 1251–1254.

[33] Cotto KC, Wagner AH, Feng YY, Kiwala S, Coffman AC, Spies G, Wollam A, Spies NC, Griffith OL, Griffith M. DGIdb 3.0: a redesign and expansion of the drug-gene interaction database. Nucleic Acids Research. 2017.10.1093/nar/gkx1143PMC588864229156001

[34] Bossy-Wetzel E, Talantova MV, Lee WD, Schölzke MN, Harrop A, Mathews E, Götz T, Han J, Ellisman MH, Perkins GA (2004). Crosstalk between nitric oxide and zinc pathways to neuronal cell death involving mitochondrial dysfunction and p38-activated K+ channels. Neuron.

[35] Rogers JM, Taubeneck MW, Daston GP, Sulik KK, Zucker RM, Elstein KH, Jankowski MA, Keen CL (1995). Zinc deficiency causes apoptosis but not cell cycle alterations in organogenesis-stage rat embryos: effect of varying duration of deficiency. Teratology.

[36] Andrews G, Wang H, Dey S, Palmiter RD. Mousezinc transporter 1 gene provides an essential function during early embryonic development. Genesis. 2004.10.1002/gene.2006715452870

[37] Gálvez-Peralta M, He L, Jorge-Nebert LF, Wang B, Miller ML, Eppert BL, Afton S, Nebert DW (2012). ZIP8 zinc transporter: indispensable role for both multiple-organ organogenesis and hematopoiesis in utero. PLoS One.

[38] Gianluca T, Roberto BC, Di CM, Andrea P, Vincenzo A, Francesca C, Mario DC (2015). Zinc in early life: a key element in the fetus and preterm neonate. Nutrients.

[39] Lamberti LM, Walker CLF, Black RE: Zinc deficiency in childhood and pregnancy: evidence for intervention effects and program responses. In Hidden Hunger. Volume 115: Karger Publishers; 2016: 125–133.10.1159/00044207927198901

[40] Prasad AS (2009). Zinc: role in immunity, oxidative stress and chronic inflammation. Current Opinion in Clinical Nutrition & Metabolic Care.

[41] Wong CP, Rinaldi NA, Ho E (2015). Zinc deficiency enhanced inflammatory response by increasing immune cell activation and inducing IL6 promoter demethylation. Mol Nutr Food Res.

[42] Siva S, Rubin DT, Gulotta G, Wroblewski K, Pekow J (2017). Zinc deficiency is associated with poor clinical outcomes in patients with inflammatory bowel disease. Inflamm Bowel Dis.

[43] Shah D, Sachdev H (2006). Zinc deficiency in pregnancy and fetal outcome. Nutr Rev.

[44] Romagnani P, Lasagni L, Annunziato F, Serio M, Romagnani S (2004). CXC chemokines: the regulatory link between inflammation and angiogenesis. Trends Immunol.

[45] Xanthou G, Duchesnes CE, Williams TJ, Pease JE (2010). CCR3 functional responses are regulated by both CXCR3 and its ligands CXCL9, CXCL10 and CXCL11. Eur J Immunol.

[46] Boyman O, Sprent J (2012). The role of interleukin-2 during homeostasis and activation of the immune system. Nat Rev Immunol.

[47] Gavins FN, Hickey MJ (2012). Annexin A1 and the regulation of innate and adaptive immunity. Front Immunol.

[48] Prasad AS (2000). Effects of zinc deficiency on Th1 and Th2 cytokine shifts. J Infect Dis.

[49] Mackay-Sim A, Dreosti IE: Olfactory function in zinc-deficient adult mice. 1989, 76:207.10.1007/BF002536382753101

[50] Horning MS, Trombley PQ (2001). Zinc and copper influence excitability of rat olfactory bulb neurons by multiple mechanisms. J Neurophysiol.

[51] Vodyanoy V (2010). Zinc nanoparticles interact with olfactory receptor neurons. Biometals.

